# Screening Hub Genes of Hepatocellular Carcinoma Based on Public Databases

**DOI:** 10.1155/2021/7029130

**Published:** 2021-10-26

**Authors:** Shan Gao, Dongjie Zhu, Jian Zhu, Lianqiang Shen, Ming Zhu, Xuefeng Ren

**Affiliations:** Department of General Surgery, The First People's Hospital of Yuhang District, Hangzhou, Zhejiang 311100, China

## Abstract

Tumor recurrence and metastasis often occur in HCC patients after surgery, and the prognosis is not optimistic. Hence, searching effective biomarkers for prognosis of is of great importance. Firstly, HCC-related data was acquired from the TCGA and GEO databases. Based on GEO data, 256 differentially expressed genes (DEGs) were obtained firstly. Subsequently, to clarify function of DEGs, clusterProfiler package was used to conduct functional enrichment analyses on DEGs. Protein-protein interaction (PPI) network analysis screened 20 key genes. The key genes were filtered via GEPIA database, by which 11 hub genes (F9, CYP3A4, ASPM, AURKA, CDC20, CDCA5, NCAP, PRC1, PTTG1, TOP2A, and KIFC1) were screened out. Then, univariate Cox analysis was applied to construct a prognostic model, followed by a prediction performance validation. With the risk score calculated by the model and common clinical features, univariate and multivariate analyses were carried out to assess whether the prognostic model could be used independently for prognostic prediction. In conclusion, the current study screened HCC prognostic gene signature based on public databases.

## 1. Introduction

Liver cancer ranks sixth of most frequent cancers and fourth of primary causes of cancer death throughout the world [1]. Hepatocellular carcinoma (HCC) (accounting for 75%-85%) is involved in primary liver cancer [2]. Hepatectomy, radiofrequency ablation, transcatheter arterial chemoembolization, liver transplantation, chemotherapy, and other strategies were applied on HCC, but its prognosis is still not optimistic [3]. About 70% of HCC patients present tumor metastasis or recurrence within 5 years after surgery [4]. Histological grade, regional invasion, distant metastasis, and other independent risk factors are closely related to recurrence and poor prognosis of HCC [5]. Nevertheless, the continuous improvement of tumor heterogeneity and molecular mechanism research have discovered more and more molecular markers of HCC, which will offer new strategies for HCC treatment.

Microarray technology and bioinformatics methods have been extensively applied to screen differentially expressed genes (DEGs) at the genomic level to help us identify HCC-related DEGs and functional pathways. In addition, gene chips can quickly detect DEGs, generate slice data, and store them in public databases, which is a reliable technique [6]. Therefore, a large number of valuable evidences can be mined for new researches based on these data. For example, more and more potential biomarkers can be mined by using public databases [7–9]. For instance, a study of Wang et al. used RNA sequencing (RNA-seq) data of clear cell renal cell carcinoma from the TCGA database to identify DEGs and 15 hub genes were found to be important in predicting the prognosis and progression of ccRCC [10]. The study of Huang et al. identified the module most related to high-level prostate cancer and revealed the hub genes within the module [11]. For HCC, the top 25% DEGs from the GSE62232 dataset were selected by Kong et al. to screen modules related to prognosis, and a protein-protein interaction (PPI) network was made to screened out 5 candidate genes including PCNA, RFC4, PTTG1, H2AFZ, and RRM1 [12].

Here, two mRNA microarray datasets and a seq dataset were obtained from the GEO and TCGA databases; then, DEGs were obtained after analysis. Later, Gene Ontology (GO) and Kyoto Encyclopedia of Genes and Protein interaction (KEGG) enrichment analyses were used to predict the DEGs involved biological functions and pathways. PPI network and Cox analysis were introduced for screening prognostic gene signature.

## 2. Materials and Methods

### 2.1. Data Download and Processing

GSE36376 (normal 193, tumor 240) and GSE76427 (normal 52, tumor 115) datasets were selected from the GEO database (https://www.ncbi.nlm.nih.gov/geo/). The platform of the both datasets was GPL10558Illumina HumanHT-12 V4.0 chip. Gene expression matrix and clinical data of HCC were accessed from the TCGA database for further validation. Differential expression analysis (∣logFC | >1, *FDR* < 0.05) was conducted by Limma package [13].

### 2.2. Enrichment Analyses of DEGs and PPI Construction

GO and KEGG enrichment analyses were carried out on DEGs using the clusterProfiler package [14] of R software. GO enrichment analysis is used to study biological significance of DEGs. KEGG pathway enrichment analysis seeks for key pathways closely related to DEGs. Thresholds are as follows: FDR < 0.05 and *P* value < 0.05.

PPI networks were constructed for DEGs by using the STRING database, respectively [15]. Then, interaction score > 0.4 was used to construct PPI networks. Cytoscape 3.7.0 was used to visualize the genes in PPI networks and to exhibit connectivity degree between genes in networks. After that, top ten genes of the number of connection nodes were selected to construct a PPI network diagram separately.

### 2.3. Prognostic Model Construction and Evaluation

Cox regression analysis was applied to construct prognostic model with “survival” R package [16]. The principal component analysis (PCA) was used to determine whether samples could be divided into different clusters based on risk score by the factoextra R package [17]. The ROC curve was plotted by the timeROC package [18].

### 2.4. Survival Analysis of DEGs

The GEPIA database can be used for individual analysis. In this study, the confirmation of expressions, overall survival (OS) analysis, and disease-free survival (DFS) analysis of the above key genes were performed using the GEPIA database, and log-rank tests were used to measure statistical significance. Survival R package [16] was used for plotting the survival curve between the high- and low-risk groups.

## 3. Results

### 3.1. Screening of Important DEGs in HCC

Two datasets (GSE36376 and GSE76427) related to HCC in the GEO database were selected. Subsequently, differential analysis was conducted on the datasets with ∣logFC | >1 and FDR < 0.05. There were 446 DEGs in the GSE36376 dataset (83 upregulated DEGs, 363 downregulated DEGs) (Figure 1(a)), while 437 DEGs were in the GSE76427 dataset (70 upregulated DEGs, 367 downregulated DEGs) (Figure 1(b)). Next, DEGs of the two datasets were intersected to obtain the shared DEGs. As shown in Figures 1(c) and 1(d), there were 24 genes of high expression and 232 genes of low expression in common. These important DEGs were selected for subsequent analysis.

### 3.2. Functional Analyses

GO analysis results revealed that 24 intersected upregulating genes were mainly concentrated in nuclear division, chromosome segregation, mitotic nuclear division, spindle organization, sister chromatid segregation, and other pathways (Figure 2(a)). KEGG analysis exhibited that these genes were mainly gathered in signaling pathways such as oocyte meiosis, cell cycle, and human T-cell virus 1 infection (Figure 2(b)). Intersected downregulating genes were mainly concentrated in small molecule catabolic process, organic acid biosynthetic process, lipid localization, lipid transport, acute inflammatory response pathway, and protein activation cascade (Figure 2(c)). These genes were in the chemical carcinogenesis, retinol metabolism, metabolism of xenobiotics by cytochrome P450, chemical carcinogenesis, complement and coagulation cascades, drug metabolism-cytochrome P450, and carbon metabolism signaling pathways (Figure 2(d)). Therefore, these DEGs may influence the progression of HCC by influencing these pathways.

### 3.3. Establishment and Analysis of PPI Networks

PPI networks were constructed, and node degree was calculated. The corresponding node degrees of top 10 hub genes were exhibited in Table 1. In Figures 3(a) and 3(b), PPI networks with upregulated and downregulated significant bias were, respectively, constructed. For better visualization, Cytoscape was used to construct the interaction diagrams of 10 highly expressed and 10 lowly expressed hub genes. It could be observed that there were interactions between these genes, indicating that the interactions may be associated with development of HCC (inhibiting or promoting the development of HCC). In addition, TOP2A and FTCD were located in the center of the diagram, so it was considered that they could be used as targets to further explore their role in HCC.

### 3.4. Hub Gene Identification and Prognostic Model Construction in HCC

20 key genes were analyzed by the GEPIA database, and it was suggested that the upregulation and downregulation of 15 genes were in accordance with this study. Both the OS curves of 13 genes and the DFS of 14 genes had biological significance. Genes with significant differences in expression analysis, OS analysis, and DFS analysis were intersected, and 11 genes (ASPM, AURKA, CDC20, CDCA5, KIFC1, NCAPG, PRC1, PTTG1, TOP2A, CYP3A4, and F9) were finally screened out as hub genes for subsequent verification (Figure 4(a)). To examine the correlation between the hub genes and prognosis status, univariate Cox analysis was introduced constructing a 10-gene prognostic signature in the TCGA dataset which was referred to as the training set (Figure 4(b)). The samples from the TCGA database were divided into the high- and low-risk groups based on the median value of risk score (Figure 4(c)). Also, the expression profile and survival status distribution of the samples were presented (Figures 4(d) and 4(e)). To examine the prediction performance, ROC curves was plotted based on the training set and validation set (GSE76427), respectively, revealing an optimal performance in the predictions (Figures 4(f) and 4(g)). In addition, PCA and survival analysis were employed for a further validation. PCA indicated that the high- and low-risk groups were obviously divided into two clusters (Figure 4(h)), and for survival analysis, patients with low risk shared a relatively optimal survival status (Figure 4(i)). To identify whether risk score could be used as an independent risk indicator, univariate and multivariate Cox analyses were conducted on the common clinical features and risk score. As the results illustrated, the prognostic model presented a robust independency (Figures 5(a) and 5(b)). Moreover, a nomogram based on the clinical features and risk score was designed for a comprehensive prediction of 1-, 3-, and 5-year-survival rates, followed by plotting the calibration curves between actual and predicted survival rates (Figures 5(c)–5(f)).

### 3.5. Examination of the Prognosis-Related Genes

To verify the prognosis-related genes (ASPM, AURKA, CDC20, CDCA5, KIFC1, NCAPG, PRC1, PTTG1, TOP2A, and CYP3A4) in HCC, the expression analysis between tumor and normal samples were presented, where we observed that the mRNA expressions of all the genes except for CYP3A4 were significantly upregulated, while CYP3A4 presented the opposite trend (Figure 6). Then, survival analyses between the high and low expressions of the genes were performed, where high expression of all the genes except for CYP3A4 gave rise to poor prognostic performances (Figures 7 and 8). To summarize, 10 prognosis-related genes showed significant difference in the terms of expression and prognostic performance.

## 4. Discussion

Main causes of HCC include chronic hepatitis virus infection, gene mutation, cell damage, alcoholic liver disease, and aflatoxin poisoning. But molecular mechanism of HCC is still less studied. An important role in HCC is cell cycle regulator [19–21]. Our study also demonstrates that the functional enrichment of DEGs is significantly upregulated in the cell cycle pathway. Cyclin D1, c-myc, RAS mutations, and cyclin D2 promoter hypermethylation are associated with HCC [22, 23]. Moreover, splicing changes of NT5E, Sulf1, and SLC39A14 were also associated with HCC [24–26]. Most HCC patients without early detection are not suitable for radical treatment, which may lead to poor prognosis of patients. Hence, potential as well as efficient markers are in urgent need. Microarray technology helps us to investigate genetic changes in HCC and identify novel biomarkers in other diseases.

Herein, DEGs were obtained from two datasets. 883 DEGs include 153 highly expressed genes and 730 lowly expressed genes. Enrichment analyses exhibited that genes with high expression were enriched in nuclear fission, mitosis, cell cycle, DNA packaging, oocyte meiotic division, folic acid synthesis, and the oocyte maturation of progesterone-mediated pathway. Lowly expressed genes were mainly in metabolic process, main immune pathways, and oxidation process, such as organic acid biosynthesis, small molecule catabolism process, lipid transport and positioning, immunoglobulin-mediated immune response, B cell-mediated response, cyclooxygenase, and P450 pathways. Cell cycle process dysregulation and mitotic cell cycle are vital in tumor development [23, 27, 28]. CDC20, one of the cell cycle regulators, was reported to serve as an oncogene [29], and in the latest study, the tumorigenesis role and the molecular mechanism of CDC20 in HCC development was pointed out as well [30]. In conclusion, GO enrichment analysis indicated that changes were mainly gathered in cell division, nuclear division, and mitosis. Changes of KEGG were in chemical carcinogenesis, glycolysis/gluconeogenesis, drug-cytochrome P450, complement and coagulation cascade, carbon metabolism, PPAR, and other signaling pathways.

In the PPI network diagrams, we selected 10 highly expressed genes and 10 lowly expressed genes as hub genes, with node degree greater than 10. Among these hub genes, the node degree of upregulated ASPM, AURKA, CCNB2, CDC20, CDCA5, NCAPG, PRC1, PTTG1, and TOP2A was 12, while the node degree of downregulated FTCD was up to 25. In these hub genes, TOP2A is confirmed to be related to early onset of HCC, shorter survival, microvascular invasion, chemotherapy resistance, and recurrence [31, 32]. Hence, it is considered a target for anticancer drugs [33–35]. HER2 and TOP2A are usually coamplified in HER2-amplified breast cancer [36]. However, the overexpression of TOP2A in HCC was not correlated with the overexpression of HER2 [37]. Besides, TOP2A can be a biomarker for diagnosis, treatment, and prognosis in lung cancer, colon cancer, and ovarian cancer [38–40]. Some clinical reports have indicated that overexpressing TOP2A is remarkably associated with shorter survival time [35, 37]. Formiminotransferase cyclodeaminase (FTCD) is expressed in every mammal, but its accumulation is highest in the liver [41]. FTCD contains two active sites (FT and CD) in different protein structures and catalyzes histidine degradation during folate metabolism [42]. Furthermore, FTCD is involved in the Golgi complex and metabolic processes [43]. FTCD is considered a candidate tumor inhibitor in HCC, which inhibits HCC by regulating cell apoptosis, DNA damage, and the phosphatidylinositol 3-kinase/Akt signaling pathway. Overexpression of FTCD inhibits cell proliferation in HCC, resulting in increased PTEN protein level in HCC cells but decreased PI3K, total Akt, and phosphorylated Akt protein levels [44]. In HCC, FTCD can also serve as a useful diagnostic biomarker to distinguish early HCC and benign tumors [45]. Herein, PPI networks showed that both TOP2A and FTCD were in the central position and had direct or indirect interactions with other genes, indicating that TOP2A and FTCD played a key role in HCC development. Later, the GEPIA database analyzed the 20 hub genes combined with expression analysis, OS analysis, and DFS analysis, and finally, 11 genes were selected for the prognostic model construction. Most of them are involved in the development of HCC and can be used as prognostic markers of HCC. An example is that upregulation of CDC20 may predict decreased OS and DFS in HCC patients [46], which is in accordance with our findings. Above studies fully demonstrate the importance of these hub genes in HCC progression.

To extract prognosis-related genes among the 20 genes from PPI network, Cox regression analysis was applied, whereby a 10-gene prognostic signature was constructed. As followed, a validation process was conducted by ROC, K-M, and PCA. Several studies have presented HCC prognostic signatures following the similar strategy [47, 48]. However, compared to the above studies, we performed a more robust HCC prognostic model based on ROC analysis results.

In summary, combining the GEO and TCGA datasets, we screened HCC prognosis-related genes, followed by examination for the prognostic model. However, the corresponding wet experiments which we are designing have not been arranged yet for practical validation.

## Figures and Tables

**Figure 1:** Identifying significant DEGs. (a, b) Volcano plots of the identified DEGs from GSE36376 and GSE76427. Black dots for nondifferentially expressed genes, and green dots along with red dots for downregulated and upregulated genes, respectively. (c, d) Intersection of upregulated and downregulated DEGs of GSE36376 and GSE76427 datasets.

**Figure 2:** Enrichment analyses for significant DEGs. (a, b) GO and KEGG enrichment analyses for upregulated DEGs. (c, d) GO and KEGG enrichment analyses for downregulated DEGs.

**Figure 3:** Top 10 hub genes in PPI networks. (a, b) Top 10 hub genes (depending on node degree) of significant highly expressed and lowly expressed DEGs, respectively. Node degree indicates the importance of genes (nodes) in the PPI network.

**Figure 4:** Screening of hub genes and constructing prognostic model. (a) Identification of hub genes, OS and DFS analyses using GEPIA. (b) Univariate cox analysis for the hub genes. (c) Arrange the samples on risk score. (d) Heat map of prognostic gene signature between the high- and low-risk groups. (e) Distribution of samples on risk score. (f, g) ROC curve of prognostic signature on 1-, 3-, and 5-year OS in the training and validation sets, respectively. (h) PCA for high- and low-risk samples (I) K-M analysis for the high- and low-risk groups; ^∗^*P* < 0.05.

**Figure 5:** Assessment of the prognostic model. (a, b) Univariate and multivariate Cox regression analyses between the risk score and clinical features. (c) Nomogram on clinical features and risk score. (d–f) Calibration curves for the predicted survival status; ^∗^*P* < 0.05, ^∗∗^*P* < 0.01, ^∗∗∗^*P* < 0.001, and ^∗∗∗∗^*P* < 0.0001.

**Figure 6:** Expression status of the prognosis-related genes.

**Figure 7:** OS survival analysis depending on the expression of prognosis-related genes.

**Figure 8:** DFS survival analysis depending on the expression of prognosis-related genes.

**Table 1:** Top 10 hub genes in PPI networks.

Gene symbol	Degree
Upregulated genes	
ASPM	12
AURKA	12
CCNB2	12
CDC20	12
CDCA5	12
NCAPG	12
PRC1	12
PTTG1	12
TOP2A	12
KIFC1	11
Downregulated genes	
FTCD	25
C8A	23
F9	23
CYP3A4	22
GPT	21
APOA5	20
FETUB	20
MBL2	20
KLKB1	19
SPP2	19

## Data Availability

The data that support the findings of this research are available on reasonable request from the corresponding author.
